The article "Diagnosis of Brain Tumor Using Light Weight Deep Learning Model with Fine-Tuning Approach" was published in 2022. Journal: Comput Math Methods Med.

# Diagnosis of Brain Tumor Using Light Weight Deep Learning Model with Fine-Tuning Approach

**DOI:** 10.1155/2022/2858845

**Published:** 2022-07-01

**Authors:** Tejas Shelatkar, Dr. Urvashi, Mohammad Shorfuzzaman, Abdulmajeed Alsufyani, Kuruva Lakshmanna

**Affiliations:** ^1^Department of Computer Science and Engineering, Dr. B. R. Ambedkar National Institute of Technology, Jalandhar 144011, India; ^2^Department of Computer Science, College of Computers and Information Technology, Taif University, P.O. Box 11099, Taif 21944, Saudi Arabia; ^3^School of Information Technology and Engineering, VIT-Vellore, India

## Abstract

Brain cancer is a rare and deadly disease with a slim chance of survival. One of the most important tasks for neurologists and radiologists is to detect brain tumors early. Recent claims have been made that computer-aided diagnosis-based systems can diagnose brain tumors by employing magnetic resonance imaging (MRI) as a supporting technology. We propose transfer learning approaches for a deep learning model to detect malignant tumors, such as glioblastoma, using MRI scans in this study. This paper presents a deep learning-based approach for brain tumor identification and classification using the state-of-the-art object detection framework YOLO (You Only Look Once). The YOLOv5 is a novel object detection deep learning technique that requires limited computational architecture than its competing models. The study used the Brats 2021 dataset from the RSNA-MICCAI brain tumor radio genomic classification. The dataset has images annotated from RSNA-MICCAI brain tumor radio genomic competition dataset using the make sense an AI online tool for labeling dataset. The preprocessed data is then divided into testing and training for the model. The YOLOv5 model provides a precision of 88 percent. Finally, our model is tested across the whole dataset, and it is concluded that it is able to detect brain tumors successfully.

## 1. Introduction

A brain tumor is a clump of uneven cells that forms a mass. Growth in this area might lead to cancerous consequences. As benign or malignant tumors develop, the pressure inside the skull will increase. Long-term brain damage and maybe death will happen as a result of this damage [1]. In India, this type of tumor affects 5 to 10 persons per 100,000 and is on the rise [2]. Considering children's brain and central nervous system, tumors are the second most common malignancy in children, accounting for around 26 percent of all malignancies.

Various advancements in the field of computer-aided diagnosis of brain tumors have been developed during the previous decade. These approaches are always available to assist radiologists who are unsure about the type of tumor they are looking at or wish to investigate further. To identify tumors, doctors utilize MRI (magnetic resonance imaging) and CT-scan (computed tomography). MRI is the most preferred technique, and hence, researchers have concentrated their efforts on MRI. A critical stage in the diagnosis of a brain tumor is segmentation. To focus on this problem, researchers are using deep learning techniques [3, 4].

The article "Diagnosis of Brain Tumor Using Light Weight Deep Learning Model with Fine-Tuning Approach" was published in 2022. Journal: Comput Math Methods Med.

Machine learning is a branch of deep learning. It employs an artificial neural network to handle difficult problems containing large volumes of information. An artificial neural network is a network that functions similarly to the brain. The word “deep” in deep learning is defined as a network with several layers. Every neuron symbolizes a function, and each link does have a certain bit of weight. The backpropagation algorithm is employed by the network by adjusting the weights. With increasing precision on complicated datasets, deep learning has changed the area of computer vision [4]. Image analysis uses a type of network called a convolutional network, which takes images as input and uses a kernel to convolve them into a picture map [5]. Deep learning models have a lot of benefits in medical imaging, including identifying critical components, pattern recognition in cell parts, feature extraction, and better outcomes for fewer datasets [6]. Transfer learning is a deep learning method in which the network's parameters (weights and biases) are taken from another network trained on a different dataset. The new network may now be trained using the transferred parameters as initialization (a process known as fine-tuning), or additional layers on top of the network can be formed and just those layers trained on the dataset of interest.

Using pretrained features on data is a common approach for neural network models [4, 7]. The network can now be developed using imported attributes as an initial process (a process known as fine-tuning), or additional layers can be placed on top of the network, with just the new layers being learned on the data of importance. Transfer learning has a number of benefits, including speeding up the data collecting process and improving generalization. It cuts down on the time it takes to train a huge dataset. In this study, we have applied YOLOv5's different variant algorithm on Brats 2020 annotated dataset to detect brain tumor location.

We used YOLO V5 to create our object detection model. The Darknet framework is utilized to maintain this model, and it provides a single network that can be used for both item categorization and prediction using bounding boxes. YOLO V5 is architecturally identical to YOLO V4, with the exception that it is built-in Python. Version 5 of YOLO is now significantly quicker and lighter. We utilized the YOLO V5 model, which was trained with the COCO dataset as a benchmark. Our unique annotated MRI pictures were used to train this model efficiently. YOLO is a single convolutional neural network, unlike other neural network-based frameworks for object identification [8, 9]. It has two fully connected layers for bounding box prediction and 24 convolutional layers for extracting information from pictures. The Darknet framework is used to build this network [10].

The article "Diagnosis of Brain Tumor Using Light Weight Deep Learning Model with Fine-Tuning Approach" was published in 2022. Journal: Comput Math Methods Med.

We have used all variations of the YOLOv5 model for brain tumor detection. The accuracy for YOLOv5s, YOLOv5n, YOLOv5m, YOLOv5l, and YOLOv5x models is 87%, 85.2%, 89%, 90.2%, and 91.2%, respectively. Lower training time, higher accuracy, and precision validate that the YOLOv5 detection model is suitable for brain tumor detection. As we have seen, there are a variety of approaches utilized in medical imaging, particularly MRI pictures of brain tumors. The algorithms for classification, segmentation, and detection were applied, but each has its own set of limitations [11, 12].

For this study, we have used a dataset from competition RSNA-MICCAI brain tumor radiogenic classification competition from Kaggle [13, 14]. The competition includes the Brats 21 dataset with a sample shown in Figure 1. The Center for Biomedical Image Computing and Analytics every year provides challenges for the researcher in terms of brain tumor analysis. The data evolves every year with improvements. The challenge has been conducted since 2013. Brats 2014-17 had a similar type of data but was discarded since it had both pre- and postoperative scans. Since 2017, the current edition of the dataset has included glioma that has been annotated by experts in order to improve the training of our model. The dataset consists of MRI images with dimensions of 240×240. The dataset consisted of images of a brain tumor in 3 types of magnetic resonance imaging scans: T1 image, T2 image, and FLAIR image.

## 2. Related Work

For the diagnosis of brain tumors, many deep learning models have been used, although object detection methods have only been used in a limited number of studies, e.g., Pereira and co-authors employed the 3D Unet model, a new deep learning model that aids in the classification of tumors according to their severity. It has considered two areas of interest, the first of which is the whole brain, and the second of which is the malignancies zone of interest [1, 15].

Neelum et al. have had a lot of success with their problem analysis since they employ pretrained models such as DesNet and Inception-v3. Concatenation of features has greatly aided the model's improvement [16]. Mohammad et al. used a small dataset of 2D images to test several machine learning algorithms such as decision trees, support vector machines, convolutional neural networks, and deep learning models such as VGG 16, ResNet, and Inception. VGG19 was the most successful model, with an F1 scope of 97.8 percent on top of the CNN framework. The author mentioned that there is a trade-off between model performance and temporal complexity. The ML approaches are simpler to use, whereas the DL methods are more efficient. The author also highlighted the need for a benchmark dataset. For tumor analysis automation, they used the algorithms FastAi and YOLOv5. However, YOLOv5 only achieves an accuracy of 85 percent. To compensate for the short dataset, they have not used any transfer learning techniques [17].

The article "Diagnosis of Brain Tumor Using Light Weight Deep Learning Model with Fine-Tuning Approach" was published in 2022. Journal: Comput Math Methods Med.

For minor health-care institutions [18], detailed research [19] on brain tumor analysis has been offered. The author conducted a poll that identified a number of issues with the methodology. They have also offered some suggestions for improving medical techniques. For bone identification, Al-masni et al. employed the YOLO model. As can be seen, the YOLO approach can produce significantly better results in medical imaging [20, 21].

Yale et al. [22] used the YOLO network to identify melanoma skin illness. Despite the fact that the test was run on a smaller dataset, the results were encouraging. The Darknet framework improves the speed of feature extraction. A better grasp of how YOLO works is still required. Kang et al. [23] suggested a hybrid model using deep features and machine learning classifiers along with the combination of several deep learning approaches with classifiers such as SVM, RBF, KNN, and others [24]. The ensemble feature has aided in the modeling of improved performance. However, the author claims that the proposed model is unsuitable for real-time medical diagnosis.

From 2015 to 2019, Muhammad et al. [17, 25] investigated several deep learning and transfer learning strategies. The author has outlined problems that must be overcome before any techniques to be used in the real world. While implementing models, researchers should pay attention to additional parameters in addition to accuracy. Some of the issues raised include the need for end-to-end deep learning models, improved run time, lower computing costs, and flexibility. The authors proposed contemporary technologies like edge computing, fog computing and cloud computing [26–28], federated learning, the GAN method, and IoT [7] as problem-solving technologies. As we have seen, there are a variety of approaches utilized in medical imaging, particularly on MRI pictures of brain tumors. The algorithms for classification, segmentation, and detection were applied, but each has its own set of limitations [11, 12].

The article "Diagnosis of Brain Tumor Using Light Weight Deep Learning Model with Fine-Tuning Approach" was published in 2022. Journal: Comput Math Methods Med.

## 3. Methodology

### 3.1. Dataset

For this study, we have used a dataset from competition RSNA-MICCAI brain tumor radiogenic classification competition from Kaggle [13, 14]. The competition includes the Brats 21 dataset with a sample as shown in Figure 1. The Center for Biomedical Image Computing and Analytics every year provides challenges for the researchers in terms of brain tumor analysis [29]. The data evolves every year with improvements. The challenge has been conducted since 2013. Brats 2014-17 had a similar type of data but was discarded since it had both pre- and postoperative scans. Since 2017, the current edition of the dataset has included glioma that has been annotated by experts in order to improve the training of our model. The dataset consists of MRI images with dimensions of 240×240. The dataset consisted of images of a brain tumor in 3 types of magnetic resonance imaging scans:

- T1 image. In these MRI scans, the fat tissue is brighter. The subcutaneous fat is brighter which is present in the bone marrow of the vertebral bodies. The cerebrospinal fluid is not highlighted as it will appear black in the scans [30]
- T2 image. This scan is opposite to that of T1 as we can see cerebrospinal fluid brightly, and the bone cortex is black in the T1 scan
- FLAIR. It is known as fluid attenuated inversion recovery. Technically, FLAIR images help in reducing the vision of fluid content so we can directly analyze the tumor

The dataset is divided into dcim images based on scan types and axial positions, such as sagittal, which is the vertical plane perpendicular to the median plane; coronal, which is perpendicular to both sagittal and coronal planes; and axial, which is perpendicular to both sagittal and coronal planes.

Brats 21 dataset also contains the mgmt value which is an enzyme in a tumor known as methylguanine methlytransferase. The mgmt value is indirectly proportional to the chemotherapy effect on patients. So, Brats 21 also provides the data about the mgmt value [31]. For brain tumor detection, we need images with exact positions for that we need to define parameters [32]. For YOLOv5 training, we clone the YOLOv5 repository which contains the YOLOv5 model for training and trained weights from the cocoa model. The YOLOv5 repository also contains the hyperparameters setting for the training of the model [33].

### 3.2. YOLOv5

The YOLOv5 model requires image input. This image needs to be preprocessed before training the model. The images taken by the model are of dimension 512. The deep learning model requires more images to train and hence has bigger dataset, and we have taken 800 images dataset. Image scaling is done on the images for better magnification of the image and detection of the tumor. The data is labeled using the makesense.ai website, which saves the labels as well as the bounding box enclosing the tumor, as well as the annotation coordinates. The labels and images are divided into test and train with the coordinates of the four vertices of the rectangular box.

The article "Diagnosis of Brain Tumor Using Light Weight Deep Learning Model with Fine-Tuning Approach" was published in 2022. Journal: Comput Math Methods Med.

The YOLOv5 model has certain advantages in its model

- The model's benefits include precise object recognition and tumor location, as well as high speed and detection accuracy
- The model is capable of detecting tiny tumor objects in photos that are noisy, hazy, or cloudy

The YOLOv5 is divided into three parts: backbone; neck; and prediction. The backbone of the YOLOv5 architecture is the Bottleneck Cross Stage Partial Darknet (BCSPD). The input images are fed to the backbone. For convolutional operations, the FOCUS module splits the input picture into four little ones and then concatenates them together. The 640×640×3 pixel picture is reduced into four smaller 320×320×3 pixel images, which are then concatenated into a 320×320×12 pixel feature map. Once 32 convolutional kernels are used, the result is a 320×320×32 feature map [34–36]. The model's CoBL module is a basic convolutional module that embodies the Conv2D + batch normalization (BN) + Leaky relu activation function. It eliminates the duplication of gradient information in CNN's optimization process and incorporates gradient changes into the feature map, decreasing input parameters and model size [37]. Two CoBL modules make up the BCSP: one residual unit and two 11 Conv2D kernels. The two CoBL modules and an adder are contained in a residual unit, and the adder adds the features of the previous CoBL module output and the features of two CoBL modules and then sends the local features to one 11 Conv2D layers. By modifying the width (w) and depth (d) of the BCSP module, the four models with varied input parameters, YOLOv5s, YOLOv5m, YOLOv5l, and YOLOv5x, may be obtained. In addition, the SPP module in the backbone interfaces with the BCSP module. The SPP module expands the network's receptive field and adds features of various scales. Second, YOLOv5 adds path aggregation network (PANet) in the neck area to improve information flow. The PANet is built on a feature pyramid network (FPN) topology, which transmits strong semantic characteristics from top to bottom. FPN layers also express significant positional characteristics from the bottom to the top. PANet also increases the transmission of low-level characteristics and the use of precise localization signals in the bottom layers. As a result, this improves the target object's position accuracy [38].

The article "Diagnosis of Brain Tumor Using Light Weight Deep Learning Model with Fine-Tuning Approach" was published in 2022. Journal: Comput Math Methods Med.

The prediction layer is also called the detection or YOLO layer, generating three different feature maps to attain multiscale prediction. However, the model can classify and detect small, medium, and large objects in the prediction layer.

The following is a synopsis of the YOLOv5 prediction process:

- Phase 1. The backbone is fed with the photos at a resolution of 640 by 640 pixels at first. The FOCUS module slices the photos after that. The feature map is sent to the second concatenation layer after performing numerous convolutional operations and two BCSP1 operations. The feature map, on the other hand, is sent to the second concatenation layer after being run once by BCSP1, twice by BCSP2, twice by convolutions, and twice by upsampling. Both of them are combined in the second concatenation layer. The 80×80 sized feature map with scale 1 is created after the BCSP2 layers and 11 convolution operations are applied
- Phase 2. The 80×80 dimension feature map from phase 1 is filtered by one 33 percent convolutional kernel in the second step and sent to the third fusion layer. In addition, one 11 convolutional kernel executes the extracted features before the second upsampling and delivers it to the third concatenation layer. The final concatenation layer then joins the two together. The 40×40 scaled feature map as scale 2 is achieved after completing the BCSP2 layer and one 1×1 convolution operation
- Phase 3. In the third phase, the convolutional kernel processes the 40×40 sized feature map from phase 2 and sends it to the fourth concatenation layer. Furthermore, one 11 convolutional kernel executes the feature map before the first upsampling and sends it to the fourth concatenation layer. Both of them are concatenated at the fourth concatenation layer. The 20×20 sized feature map as scale 3 is then created using the BCSP2 layer and the 11 convolution procedure
- Phase 4. Finally, the feature maps of various sizes in scales 1 to 3 (i.e., 80×80, 40×40, and 20×20) are enhanced for recognizing tumor objects of various sizes using regression bounding boxes (BB). As a result, each feature map is predicted to have three regression bounding boxes at each position, resulting in three (80×80, 40×40, 20×20) =25200 regression bounding boxes. Finally, as a final tumor detection outcome, the model's anticipated output with BB is displayed

The MSCOCO dataset has 80 preset object classes, and the YOLOv5 model was trained on it. The anticipated output tensor (POT) dimensions are 3 (5 + 80) = 255 where “3” signifies each grid cell prediction's three bounding boxes (BB), “5” specifies each prediction box's coordinates (xo, yo, w, and h) and confidence score (CS), and “80” denotes the predetermined item class (CL). As a result, we will need to tweak the YOLOv5 model's classifier. As a result of Equation (2), the projected output tensor (POT) dimension in our situation is 3 (5 + 2) = 21 [39].

The article "Diagnosis of Brain Tumor Using Light Weight Deep Learning Model with Fine-Tuning Approach" was published in 2022. Journal: Comput Math Methods Med.

For training our model, we have used the Google Colab environment. Once the dataset is preprocessed, we feed the training data to the pretrained model along with its hyperparameters provided by the YOLOv5 researchers for better results. In this research, we have used all the YOLOv5 variations which are available to get an in-depth analysis of the YOLOv5 model.

## 4. Evaluation Metrics

True positives (TP), false positives (FP), true negatives (TN), and false negatives (FN) are four important outcomes used to assess the efficacy of the proposed brain tumor classification and detection system. The performance of the proposed system is calculated using the following metrics: Accuracy determines the ability to correctly discriminate between different types of brain tumors [40]. The proportion of true positive and true negative occurrences in all studied cases is computed using the formula below to establish a test's accuracy.

A true positive (TP) is when the model predicts the positive class properly. A true negative (TN), on the other hand, is a result in which the model properly predicts the negative class. A false positive (FP) occurs when the model forecasts the positive class inaccurately. A false negative (FN) is an outcome in which the model forecasts the negative class inaccurately. Equation (1) has formula for accuracy, Equation (2) shows for precision, and Equation (3) represents recall. F1 formula as shown in Equation (4) is derived from precision and recall:

(1) $$\begin{array}{c} \text{Accuracy}=\frac{\text{TP}+\text{TN}}{\text{TP}+\text{TN}+\text{FP}+\text{FN}}, \end{array}$$

(2) $$\begin{array}{c} \text{Precision}=\frac{\text{TP}}{\text{TP}+\text{FP}}, \end{array}$$

(3) $$\begin{array}{c} \text{Recall}=\frac{\text{TP}}{\text{TP}+\text{FN}}, \end{array}$$

(4) $$\begin{array}{c} \text{F}1=\frac{2*\text{Precision}*\text{Recall}}{\text{Precision}+\text{Recall}}=\frac{2*\text{TP}}{2*\text{TP}+\text{FP}+\text{FN}}. \end{array}$$

## 5. Proposed Model

We will be using the state-of-the-art model YOLOv5, as previously stated. COCO (Microsoft Common Objects in Context) dataset provided the pretrained weights. This parameter is used for fine tweaking. The BRat 2020 dataset is used to train the model. Patients' 3D scans are used to input the model. We use the test picture to obtain information about the tumor once the model has been trained. Using pretrained parameters on a dataset is a common approach in deep learning models [15]. The new network can now be trained using the transferred parameters as initialization (a process known as fine-tuning as shown in Figure 2), or additional layers can be built on top of the network, with only the new layers being trained on the dataset of interest. Transfer learning has a number of advantages, including speeding up the data collection process and improving generalization. In Figure 3, we can see we have input the preprocessed dataset along with pretrained weights and hyperparameter. The data is evaluated according to the model with various operations performed in the head, neck, and prediction phase of the YOLOv5 model. It cuts down on the time it takes to train a huge dataset.

The article "Diagnosis of Brain Tumor Using Light Weight Deep Learning Model with Fine-Tuning Approach" was published in 2022. Journal: Comput Math Methods Med.

Before we train the model with the YOLO model, we need to do some preprocessing. The tumor must be designated with a box region. This may be accomplished by utilizing a tool that produces a bounding box around the image's item of interest. We can utilize the NVIDIA transfer learning toolbox for transfer learning, and we can feed the COCO dataset because it supports the YOLO architecture. This fine-tunes our model and compensates for missing or unlabeled data. Following that, we can use our model to train our Brats dataset. Google Colab, which provides 100 GB of storage, 12 GB of RAM, and GPU support, was used for development. The creators of YOLOv5 have made their training results accessible on the COCO dataset, which we may download and utilize for our own model. We need a labeled dataset for training to apply the YOLOv5 method to our model, which is available in the Brats dataset.

We will freeze several layers and put our own layer on top of the YOLO model for better results on the Brats dataset since we need to train it for better results on the Brats dataset. We will utilize the YOLOv5n model since we require a model that takes up less space. On the COCO dataset [13, 41], the YOLOv5 model gives us a mean average accuracy score of 72.4 and a speed of 3136 ms, as stated in the official repository. The key benefit of this model is that it is smaller and easier to produce than the prior YOLO model, and it is 88 percent smaller. At 140 frames per second, this model can process pictures. COCO (Microsoft Common Objects in Context) dataset provided the pretrained weights. This parameter is used for fine tweaking. The Brats 2020 dataset was used to train the model. We will use the YOLOv5 nano model in this case since it has a smaller architecture than the other models, and our major concern is model size. In comparison to the other models, the YOLO model has a significantly smaller 1.9 M params. To be able to do brain scans, our model requires a specific setup. We do different treatments on the data, ranging from scaling to masking, because the scanned data of Brats is complicated.

The article "Diagnosis of Brain Tumor Using Light Weight Deep Learning Model with Fine-Tuning Approach" was published in 2022. Journal: Comput Math Methods Med.

Because the image data is saved in different formats with various types of scans such as FLAIR, T1, and T2, it is critical to handle the dataset according to our model's familiarity. Patients' scans are input into the model. We utilize the dice score, jaccard score, and map value to evaluate the outputs of our model, but our primary focus is on the model's speed in order to improve its usefulness. The dataset has already been partitioned for training and testing purposes. There are around 360 patient scans for training and 122 patient scans for testing in our dataset. We may test the network using the YOLOv5 models' yml file for our specific setup. The classification has been set to three because we only have three classes. Our parameters in the backbone or head of our model must also be supplied to multiple convolution layers. The test picture dataset is fed to the models once the model has been trained. When compared to segmentation models, the predicted output of the proposed model must be close to a dice score of 0.85. In comparison to the previous models, this model uses less storage and processes the Brats dataset faster.

## 6. Experimental Results and Discussions

We have trained our model for different YOLOv5 variations. The YOLOv5 version includes YOLOv5s, YOLOv5n, and YOLOv5m. As we have trained from 0-50 epochs, this needs to be implemented according to lesser epoch data to check if our model is able to adapt according to lesser time requirement.  Figure 4 shows the accuracy curves for YOLOv5s, YOLOv5m, and YOLOv5l, using the final picture dataset. The accuracy rate is initially quite low in all models, as shown in Figure 4, but it increases when the epochs are increased. Furthermore, the precision rate of the YOLOv5s model is from 75 to 85 percent, while the rates of the YOLOv5m and YOLOv5l models range from 78 to 89 percent and 83 to 95 percent, respectively. As a consequence, the YOLOv5l model outperforms the other two models in terms of benign and malignant tumor classification and prediction. Recall, on the other hand, refers to a model's capacity to recognize all relevant tumor classifications. It is also worth noting that as the number of epochs grows, so does the recall rate. Furthermore, the YOLOv5s model has a recall rate ranging from 80 percent to 90 percent, while the YOLOv5m model has a rate ranging from 85 to 95 percent, and the YOLOv5l model has a rate ranging from 88 to 98 percent. As a result, the YOLOv5l model outperforms the other two models in terms of target tumor categorization and prediction. In addition, for all models, the mean average precision (mAP) is calculated. The mAP of the YOLOv5l model is higher than that of the YOLOv5m and YOLOv5s models, as can be shown in Table 1.

The article "Diagnosis of Brain Tumor Using Light Weight Deep Learning Model with Fine-Tuning Approach" was published in 2022. Journal: Comput Math Methods Med.

### 6.1. Performance

The impact of input dimensions on overall performance is shown in Table 1. The YOLOv5x variant generated the greatest mAP of 91.2% from the estimated findings from the test dataset. YOLOv5l came in second with 90.2%. Surprisingly, the YOLOv5n model did not improve on the YOLOv5s model. YOLOv5x had the greatest mAP, the accuracy of 89.1%, and RE of 90.4% in terms of total performance. With 85.2%, YOLOv5n had the lower mAP. However, as precision and complexity improve, the time required rises. The YOLOv5s model, which takes roughly 40 minutes to train for 50 epochs, requires the least amount of time. We examine different detection algorithms used for brain tumor analysis in Table 2. Faster R-CNN, as shown in Table 2, has worse accuracy than the other models, despite having greater weight and training time. YOLOv4 has a good accuracy score; however, it gives somewhat more weight to smaller models than YOLOv5. YOLOv5m produces the most consistent output with the best weight-to-accuracy ratio. After training our model, we are able to detect a tumor on any input image as shown in Figure 5.

## 7. Conclusion

In the proposed study, we have applied YOLOv5's different variant algorithm on Brats 2020 annotated dataset to detect brain tumor location. We were able to achieve 82-92 percent accuracy for the YOLO variant in which the YOLOv5l model provides us with the best accuracy than YOLOv5n and YOLOv5s. It was observed that the object detection model on brain tumor analysis gives slightly lesser accuracy than the classification and segmentation model. But we have also observed a substantial decrease in the training time and size of the model. We have also observed that while using the object detection model, there is a trade-off between the accuracy of our model with a combination of training time and model complexity. We have observed that in the YOLO model, the increase in complexity largely affects the training time, but there is an increase of about 5-6 percent in accuracy.

## 8. Future Scope

In the future, the accuracy of YOLOv5 smaller version models can be increased with further experimentation, and some additional research can be performed to decrease the trade-off between the accuracy and complexity of the model.

The article "Diagnosis of Brain Tumor Using Light Weight Deep Learning Model with Fine-Tuning Approach" was published in 2022. Journal: Comput Math Methods Med.

## Figures and Tables

**Figure 1:** Brats21 dataset.

**Figure 2:** Fine-tuned YOLOv5 model.

**Figure 3:** YOLOv5 model.

**Figure 4:** Accuracy curves for YOLOv5s, YOLOv5m, and YOLOv5l.

**Figure 5:** Brain tumor detection using proposed model.

**Table 1:** YOLOv5 implementation analysis.

Model	Weight	mAP
Faster R-CNN [42]	200 mb	77.60
YOLOv4-tiny	33.2 mb	88.98
YOLOv5s	17 mb	87
YOLOv5n	12 mb	85.2
YOLOv5m	41 mb	89
YOLOv5l	90 mb	90.2
YOLOv5x	168 mb	91.2

**Table 2:** YOLOv5 comparison analysis.

Model	Weight	Precision	Times required (minutes)	Recall	mAP
YOLOv5s	17 mb	82.9	82.9	83	87
YOLOv5n	12 mb	81.5	81.5	82	85.2
YOLOv5m	41 mb	85.2	85.2	87.4	89
YOLOv5l	90 mb	88.2	88.2	86.2	90.2
YOLOv5x	168mb	89.1	190.1	9	91.2

## Data Availability

The data can be provided based on the request from the corresponding author.
